# Finite Element Analysis of a Novel Anterior Locking Plate for Thoracolumbar Burst Fracture

**DOI:** 10.1155/2021/2949419

**Published:** 2021-10-11

**Authors:** Pengcheng Ren, Xiaodong Cheng, Chongyao Lu, Haotian Wu, Shuangquan Yao, Sidong Yang, Zhaohui Song

**Affiliations:** ^1^Department of Orthopedic Surgery, The Third Hospital of Hebei Medical University, No. 139 Ziqiang Road, Qiaoxi District, Shijiazhuang 050051, China; ^2^Key Laboratory of Biomechanics of Hebei Province, Shijiazhuang, Hebei, China; ^3^Australian Institute for Bioengineering and Nanotechnology, The University of Queensland, Australia

## Abstract

**Purpose:**

The finite element analysis method was used to explore the biomechanical stability of a novel locking plate for thoracolumbar burst fracture fusion fixation.

**Methods:**

The thoracolumbar CT imaging data from a normal volunteer was imported into finite software to build a normal model and three different simulated surgical models (the traditional double-segment fixation model A, the novel double-segment fixation model B, and the novel single-segment fixation model C). An axial pressure (500 N) and a torque (10 Nm) were exerted on the end plate of T12 to simulate activity of the spine. We recorded the range of motion (ROM) and the maximum stress value of the simulated cages and internal fixations.

**Results:**

Model A has a larger ROM in all directions than model B (flexion 5.63%, extension 38.21%, left rotation 46.51%, right rotation 39.76%, left bending 9.45%, and right bending 11.45%). Model C also has a larger ROM in all directions than model B (flexion 555.63%, extension 51.42%, left rotation 56.98%, right rotation 55.42%, left bending 65.67%, and right bending 59.47%). The maximum stress of the cage in model A is smaller than that in model B except for the extension direction (flexion 96.81%, left rotation 175.96%, right rotation 265.73%, left bending 73.73%, and right bending 171.28%). The maximum stress value of the internal fixation in model A is greater than that in model B when models move in flexion (20.23%), extension (117.43%), and left rotation (21.34%).

**Conclusion:**

The novel locking plate has a smaller structure and better performance in biomechanical stability, which may be more compatible with minimally invasive spinal tubular technology.

## 1. Introduction

Traditional anterior surgery is recommended for patients with nerve compression from the front, the intact posterior ligamentous complex (PLC), and incomplete spinal cord injury [1–3]. This procedure can perform the decompression and fusion operation of the anterior middle column under direct vision to provide a better nerve decompression effect and fusion stability [4]. However, it is full of controversy due to the complicated surgical approach and many postoperative complications [5–8]. With the development of spine devices, anterior minimally invasive spinal tubular technology, such as anterior lumbar interbody fusion (ALIF), oblique lateral interbody fusion (OLIF), and direct lateral interbody fusion (DLIF), which requires smaller incisions and avoids excessive approach-related injury while allowing rapid recovery [9, 10], has become more popular in recent years. This technique is mostly used in the treatment of intervertebral discs, but is rarely used in the treatment of vertebral body fusion for spinal fractures [11–13].

In the course of clinical treatment, we try to use minimally invasive tubular technology to treat the thoracolumbar burst fractures that require anterior decompression and fusion. However, the traditional anterior fixation instrument cannot well cooperate with the channel technology to perform the operation. Based on this feature, we designed and invented an internal fixation device (Figure 1) (Patent No., ZL 201810805552.8) that can meet the requirements of a smaller size, a more concise connection method, and provide better stability.

In order to evaluate the biomechanical properties of the novel plate, this experiment uses finite element analysis to compare the novel fixation instrument with the traditional double-segment fixation instrument (TDFI). By analyzing statistics of the range of motion (ROM) and the maximum stress value of the simulated cages and internal fixations, we try to appraise the biomechanical stability of the novel instrument in single-segment fixation instrument (NSFI) and double-segment fixation instrument (NDFI).

## 2. Materials and Methods

### 2.1. Novel Plate Design

The appearance of the new plate we designed is shown in Figure 1. The material of the new internal fixation is titanium alloy, the shape of the plate is “I,” and its arc is the same as that of the side-wall of the vertebral. There are 3 holes on both sides of the plate for locking screws. When inserting the locking screw, the screw should be close to the endplate and perpendicular to the sagittal axis of the vertebral body. At this time, the plate and screws can support the endplate. The screw is designed as a cortical locking screw with a diameter of 3.5 mm—while the value of traditional screw diameter is about 5.5 mm—and the length span is 5 mm. The novel plate is designed in different sizes, and the width is about 26 mm and the length 70 mm, for various patients to choose. Compared with the larger screw diameter in the traditional anterior system, the newly designed internal fixation apparatus reduces the screw diameter, which can complete the screw installing with only a small amount of bone remaining in the injured vertebra and achieve the goal of single-segment or double-segment fusion fixation.

### 2.2. Building a Normal Finite Element Model

We selected a 25-year-old male volunteer who was in good health and had never got spinal disease or pain and screened by X-ray. After explaining the risks and benefits of CT scan in detail, the volunteer signed the informed consent. On March 13, 2019, the volunteer's T12-L5 vertebral was scanned by 64-slice spiral CT (Siemens, Erlangen, Germany) in the CT room of the Third Hospital of Hebei Medical University. The tube current of the machine used is 200 mA, the tube voltage is 120 kV, the slice thickness is 1 mm, the interlayer spacing is 1 mm, and the image data output is in DICOM (Digital Imaging and Communications in Medicine) format.

The DICOM format image data was imported into the interactive medical imaging control system Mimics17.0. The threshold segmentation was used to remove the other structures except the T12-L4 vertebral body; then, a 3D spine model of the T12 to L4 was created. These models were imported into the reverse engineering software Geomagic Studio 12.0, and the obvious defects of the vertebral body were removed using smoothing and denoising. The intervertebral disc structures of T12-L1, L1-L2, L2-L3, and L3-L4 were designed and established by using UG NX9.0 software in which the nucleus pulposus occupied 44% of the area of the intervertebral disc (Figure 2). The 3D spine model was imported into the Hypermesh program to divide the 3D structure into a mesh model including 441135 nodes and 975423 elements. Finally, the divided model was imported into the Abaqus finite element analysis software to establish ligament structures around the model and named M0 (Figure 3), including the anterior longitudinal ligament, posterior longitudinal ligament, ligamentum flavum, interspinous ligament, supraspinous ligament, and intertransverse ligament. Each structure was assigned material properties (Table 1) [14, 15], including elastic modulus and Poisson's ratio.

### 2.3. Building Anterior Depression Model of the L2

According to the characteristic of the anterior approach, the completed 3D thoracolumbar model was imported into the UG NX9.0 software to build three simulated depression models. They were divided into two forms: (1) the upper 1/2 bone of the L2 vertebrae and the adjacent intervertebral disc were removed to meet the single-segment decompression and fusion surgery, and this model only created one; (2) both L2 vertebrae and all the adjacent intervertebral discs were removed to meet the double-segment decompression and fusion surgery, and two models of this type were established.

### 2.4. Building Model of the Cage and Internal Fixation Devices

The cage and internal fixation devices were built by the UG NX9.0 software (Figure 4). The material of all apparatuses was titanium alloy, and each part connected with a locked form. All the internal fixation devices were placed on the left side of the spine models. (1) The data of the traditional anterior two-segment fixation system was provided by Double-Medical Technology Co., Ltd. The diameter of the vertebral screw was 5.5 mm, and the length was 50 mm; the diameter of the connecting rod was 5.5 mm, and the length was 70 mm and 85 mm; the width of the double hole gasket was 4 mm, and the height was 8.5 mm. (2) The data of the novel two-segment plate was designed by ourselves, the length of the plate was 78 mm, and the width of the plate was 26 mm. The screw diameter was 3.5 mm, and the length was 45 mm. (3) The length of the novel single-segment plate was only 20 mm shorter than that of the double-segment plate, while the other parameters remained unchanged. (4) Titanium cage data was provided by Double-Medical Technology Co., Ltd. In order to apply to different fusion segments, we created three cage models in two types that only had differences in length: two cages with 40 mm and one cage with 18 mm. Their diameters were 24 mm, and thicknesses were 1.5 mm. Finally, the Hypermesh program was used to mesh all apparatuses: the traditional fixation system had 28491 nodes and 127158 elements; the novel two-segment plate had 8095 nodes and 27046 elements; the novel single-segment plate had 7773 nodes and 26400 elements; the bigger cage had 3585 nodes and 8778 elements but smaller 2230 nodes and 5957 elements.

### 2.5. Establishing Different Surgical Models in Finite Element Software

The meshed models in Hypermesh were imported into the finite element software Abaqus to give material properties (Table 1), including elastic modulus and Poisson's ratio. The two-segment fixation with the traditional instrument was named model A, the two-segment fixation with the novel plate was named model B, and the single-segment fixation with the novel plate was named model C (Figure 5).

### 2.6. Setting Up Loads and Boundaries

The boundaries and loads were set to simulate spinal movement using the finite element software Abaqus. The boundaries were defined as the lower part and back of the L4 vertebrae that were set to be fixed. The rotation of the spine around the *X*, *Y*, and *Z* axes was defined as the flexion-extension, lateral bending, and rotation of the spine. According to normal human body weight bearing and previously published literature [16–18], an axial load of 500 N and a torque of 10 Nm are uniformly applied to the T12 endplate.

### 2.7. Evaluation Index

It analyzed the spinal motion range of the thoracolumbar spine in 6 different directions and the maximum von Mises stress of cages and internal fixations in the three models. No statistical analysis was performed in this study as only one subject was modeled.

## 3. Results

### 3.1. Results of Model Validity

In order to verify the validity of the model, we applied 150 N axial pressure and 10 Nm torque on the upper surface of the T12 vertebrae to measure the ROM of the model in all directions. The measured range of motion of the normal model under various working conditions is similar to the results of previous biomechanical studies (Table 2) [16, 17, 19], which proves the validity of the finite element model established in this study.

### 3.2. The Results of Range of Motion

The upper surface of T12 was uniformly applied 500 N axial load and 10 Nm torque to simulate spinal motion (Figure 6), and the ROM of the simulated models was recorded (Figure 7). The ROM of the three simulated models in all directions is smaller than that of the normal model. Among the three simulated models, model C has the largest range of motion in six directions, and model B has the smallest range of motion in six directions. Compared with model B, model A has an increase of 5.63% in flexion, 38.21% in extension, 46.51% in left axial rotation, 39.76% in right axial rotation, 9.45% in left bending, and 11.45% in right bending. Compared with model B, model C has an increase of 555.63% in flexion, 51.42% in extension, 56.98% in left axial rotation, 55.42% in right axial rotation, 65.67% in left bending, and 59.47% in right bending.

### 3.3. The Maximum von Mises Stress of Each Internal Fixation and Cage

The maximum von Mises stress of the cages in each model in different directions of motion is shown in Figure 8. When bending on the left side, each simulated surgery model shows that the stress of the cage is the smallest. We chose model A and model B to appraise the maximum von Mises stress because they only have differences in the internal fixation device. Except in the extension direction, the stress in the other motion directions of model A is much greater than the stress of the cage in model B. The maximum von Mises stress of the cage in model A decreases by 29.11% in the extension but increases by 96.81% in the flexion, 175.96% in the left axial rotation, 265.73% in the right axial rotation, 73.73% in the left bending, and 171.28% in the right bending.

The maximum von Mises stress of the internal fixation devices in each model in different directions of motion is shown in Figure 9. In the flexion, extension, and left axial rotation, the maximum von Mises stress of model A is larger than that of the model B by 20.23%, 117.43%, and 21.34%. In the right axial rotation, left bending, and right bending, the maximum von Mises stress of model A is reduced by 27.38%, 20.77%, and 7.54% compared with the model B.

## 4. Discussion

We designed a finite element experiment to compare the effects of novel plate and traditional internal fixation device on spinal stability and range of motion after surgical fixation. The results show that the novel plate provides better postfusion stability, and the reduction of fusion segments has a smaller effect on spinal mobility. Meanwhile, the new internal fixation device can better disperse the stress to avoid internal fixation stress concentration.

Anterior channel technology is mostly used in thoracolumbar degenerative diseases to treat intervertebral disc lesions and complete intervertebral fusion [20, 21], but it is rarely used in thoracolumbar burst fractures. Based on the concept of minimally invasive, we use channel technology to perform anterior decompression and fusion treatment for burst fracture patients with complete PLC and neurological impairment. In the course of treatment, we found that nerve decompression can be completed with only a portion of the injured vertebrae bone removed. However, due to the cumbersome connection of the anterior screw rod internal fixation device and the relatively large screw diameter, it cannot be well matched with the channel technology to complete the fixation with little bone remaining in the injured vertebra. In view of these considerations, we newly designed a more compact and convenient device to match the working channel to achieve the purpose of obtaining maximum stability while fixing fewer segments. The “raft support” [22] concept used in the treatment of the long tubular bone metaphysis is integrated into the newly designed plate. The diameter of the screw is reduced while the number of screws is increased, so that the screws are arranged in a plane at both sides of the plate, which can support the endplates.

In this experiment, the range of motion of the three simulated models is less than that of the normal model. Previous literature has shown that no matter what kind of surgical fixation method, it will have different degrees of influence on the mobility of the spine [23, 24], and the results in this experiment also reflect similar problems. A comparison between model A and model B shows that only the internal fixation method is different, so the larger the movement range, the worse the stability of the internal fixation. The results that the novel locking plate method has a smaller ROM explain the locking manner of the novel plate, which makes the screw and the plate integrated, is simpler and more reliable than the traditional nail-rod press-fit fixing method. Spinal fusion surgery will cause changes in the pressure in the intervertebral discs of adjacent segments. Over time, the intervertebral discs of adjacent segments may undergo metamorphosis, and there is a risk of developing adjacent segment disease (ASD) [25]. Biomechanical studies of simulated lumbar fusion surgery have shown that the pressure in the adjacent intervertebral discs of the fusion segment will increase, and the increase in pressure is positively correlated with the number of fusion segments [26, 27]. The longer the fusion segment, the more likely it is to develop ASD. The newly designed plate reduces the diameter of the screw which requires less residual bone in the injured vertebra so it might reduce the fusion segment to decrease the incidence of ASD.

We also measured the maximum von Mises stress of each internal fixation and cage to judge the support effect of different internal fixation devices on the spine. The cage is located between the two vertebral bodies, and its force can reflect the amount of stress shared by the internal fixation. Our results of the maximum stress of the cage indicate that the new plate bears more stress than the traditional device, because the screws are arranged in a plane to provide planar support to the endplate, which provides stronger stability than the traditional linear support structure with two nails. Maintaining a stable state can also provide a better mechanical environment for the growth and fusion of bone tissue. Although the new plate bears more stress, the maximum stress value on the internal fixation is smaller than that of the nail-rod system in the movement direction of flexion, extension, and left axial rotation. In the new plate system, the screw and the plate form a whole through a locking structure, which disperses the stress on the screw-plate structure and is not prone to stress concentration, thereby reducing fatigue break of the internal fixation.

There are also some shortcomings in the research. Although the finite element software can simulate movement of spine and measure the stress on the internal fixation, it only loads the force in six directions and still cannot fully simulate all the characteristics of the human body in which the movement of the spine is produced by the contraction of different muscles. Various material properties are also assigned with reference to different documents, which may be different from the real organization. The method of finite element analysis will have personal errors when the model is established, and some structures will be different from the real spine condition. Moreover, maximum stress experiments and fatigue experiments are required to further test the properties of the plate. If necessary, we will further improve the device because the new plate is still in the experimental stage.

## Figures and Tables

**Figure 1:** Preliminary design of the novel plate appearance. (a) The position of the plate on the spine mold. (b) Screws position under transverse section. (c) The shape of the novel plate and screws.

**Figure 2:** The normal T12-L4 thoracolumbar model designed in UG NX software. (a) Normal model anteroposterior view. (b) Normal model lateral view.

**Figure 3:** The normal T12-L4 thoracolumbar model (M0) in finite element software Abaqus. Imported the meshed 3D model into the finite element software, build ligaments model, and assigned material properties.

**Figure 4:** The models of different surgical protocols designed in UG NX software. (a) Anteroposterior and lateral view of the traditional double-segment screws fixation system. (b) Anteroposterior and lateral view of the novel double-segment plate fixation system. (c) Anteroposterior and lateral view of the novel single-segment plate fixation system.

**Figure 5:** The models of different surgical protocols in finite element software Abaqus. Imported the meshed 3D model into the finite element software, built ligaments model, and assigned material properties. (a) Anteroposterior view of the traditional double-segment screws fixation system (model A). (b) Anteroposterior view of the novel double-segment plate fixation system (model B). (c) Anteroposterior of the novel single-segment plate fixation system (model C).

**Figure 6:** Movement of three models under different working conditions. Apply 500 N axial load and 10 Nm torque to the endplate on T12 and observe the range of motion of the models in all directions. I.-III. represent model A, model B, and model C; i.-vi. represent different directions of motion, including flexion, extension, left axial rotation, right axial rotation, left lateral bending, and right lateral bending.

**Figure 7:** The results of range of motion.

**Figure 8:** The maximum von Mises stress of cages.

**Figure 9:** The maximum von Mises stress of internal fixations.

**Table 1:** Material properties of the finite element models.

Structures	Elastic modulus (MPa)	Poisson ratio	Sectional area (mm^2^)
Cortical bone	12000	0.3	
Cancellous bone	100	0.3	
Annular fiber	450	0.45	
Nucleus pulposus	1	0.49	
Anterior longitudinal ligament	7.8	0.3	49
Posterior longitudinal ligament	10	0.3	30
Ligamentum flavum	15	0.3	40
Interspinous ligament	10	0.3	70
Supraspinous ligament	10	0.3	70
Intertransverse ligament	10	0.3	2
Internal fixation devices	110000	0.3	

**Table 2:** Comparison between the normal spine model and models from previous studies.

	ROM (°)			
	Results	Yamamoto et al. [16]	Pflugmacher et al. [17]	Basaran et al. [19]
Flexion	5.46	5.8 ± 0.6	5.3 ± 1.0	4.5 ± 0.9
Extension	4.71	4.3 ± 0.5	5.7 ± 1.0	4.5 ± 0.9
Left bending	4.67	5.2 ± 0.4	4.3 ± 0.6	4.2 ± 0.8
Right bending	4.55	4.7 ± 0.4	4.3 ± 0.6	4.2 ± 0.8
Left rotation	1.53	2.6 ± 0.5	2.1 ± 0.5	2.3 ± 0.6
Right rotation	1.88	2.0 ± 0.6	2.1 ± 0.5	2.3 ± 0.6

## Data Availability

All data analyzed during this study are included in this article.

## Abbreviations

PLC: Posterior ligamentous complex
TDFI: The traditional double-segment fixation instrument
NSFI: The novel instrument in single-segment fixation instrument
NDFI: The novel instrument in double-segment fixation instrument
ROM: Range of motion
3D: Three dimensional
CT: Computed tomography
DICOM: Digital imaging and communications in medicine
ASD: Adjacent segment disease.
